The article "Seasonal correlation of aerosols with soil moisture, evapotranspiration, and vegetation over Pakistan using remote sensing" was retracted in 2024. Reasons: unreliable results or conclusions; a breach of policy by an author; concerns about the authorship.

# Seasonal correlation of aerosols with soil moisture, evapotranspiration, and vegetation over Pakistan using remote sensing

**DOI:** 10.1016/j.heliyon.2023.e20635

**Published:** 2023-10-04

**Authors:** Uzma Basharat, Salman Tariq, Muhammad Nawaz Chaudhry, Muhammad Khan, Ephraim Bonah Agyekum, Wulfran Fendzi Mbasso, Salah Kamel

**Affiliations:** a Lahore School of Economics, Pakistan; b Remote Sensing, GIS and Climatic Research Lab (National Center of GIS and Space Applications), Centre for Remote Sensing, University of the Punjab, Lahore, Pakistan; c Department of Space Science, University of the Punjab, Lahore, Pakistan; d Department of Nuclear and Renewable Energy, Ural Federal University Named After the First President of Russia Boris, 19 Mira Street, Ekaterinburg, 620002, Yeltsin, Russia; e Laboratory of Technology and Applied Sciences, University Institute of Technology, University of Douala, PO Box: 8698, Douala, Cameroon; f Department of Electrical Engineering, Faculty of Engineering, Aswan University, 81542, Aswan, Egypt

**Keywords:** Aerosol optical depth, Angstrom exponent, Soil moisture, Evapotranspiration, Normalized difference vegetation index

## Abstract

Aerosols have a severe impact on the Earth's climate, human health, and ecosystem. To understand the impacts of aerosols on climate, human health, and the ecosystem we must need to understand the variability of aerosols and their optical properties. Therefore, we used Aqua-MODIS retrieved aerosol optical depth (AOD) (550 nm) and Angstrom exponent (AE) (440/870) data to analyze the Spatio-temporal seasonal variability of aerosols and their relationship with different meteorological parameters over Pakistan from 2002 to 2021. High (>0.5) AOD values were observed during the summer season and low (<0.8) in the spring season. AE values were observed to be high (>1) in the northern regions of Pakistan indicating the dominance of fine mode particles during the winter season. Moreover, AOD showed a positive correlation with Relative Humidity (RH), Evapotranspiration, Wind speed (WS), and Temperature. On the other hand, it showed a negative correlation with Soil moisture (SM), Normalized difference vegetation index (NDVI), and precipitation over Pakistan. Therefore, considering the outcomes of this study will help policymakers to understand the spatiotemporal variability of aerosols and their seasonal correlation with different meteorological parameters.

## 1 Introduction

Aerosols are particles suspended in the air [1,2]. Aerosols are produced by both natural (i.e dust originating from deserts, forest fires, and volcanic eruptions) and anthropogenic activities (burning of crop residue and fossils) within the region [[3], [4], [5]]. Aerosols are responsible for producing greenhouse gases that can cause global warming [6]. Aerosols in the atmosphere impact the quality of air, the hydrological cycle, precipitation rate (PR), and energy balance [7,8]. They cause the formation of fog, clouds, and smog in the atmosphere [9,10].

The article "Seasonal correlation of aerosols with soil moisture, evapotranspiration, and vegetation over Pakistan using remote sensing" was retracted in 2024. Reasons: unreliable results or conclusions; a breach of policy by an author; concerns about the authorship.

The weather conditions and the emission of aerosols from local sources make up the concentration of aerosols in a particular region. The increased number of aerosols in Asia is due to an increase in traffic, urbanization, and industrialization [[11], [12], [13]]. The diverse change in global climate patterns due to cooling and warming of the atmosphere is because of aerosols present in the atmosphere. However, having an understanding of aerosols and their interaction has become tough due to the variations in their distribution within the atmosphere [14]. Lensky and Rosenfeld [15] studied the effect of convective clouds and rainfall on aerosols. Grypspeerdt et al. [16] investigated global climate change due to anthropogenic activities.

Tariq et al. [17] analyzed the Spatiotemporal distribution and trend analysis of Aerosol Optical Depth (AOD) over South Asia from September 2002 to December 2020. Sreekanth et al. [18] reported that AOD increased in the monsoon and summer seasons from 2002 to 2011 in India. Duan et al. [19] similarly analyzed the variability of absorbing aerosols over three provinces in China. Su et al. [20] also analyze the optical and physical properties of aerosols in northern China. Khan et al. [21] reported a high concentration of aerosols during 2021 in Pakistan using OMI-retrieved UVAI data from 2004 to 2021. Tariq et al. [22] similarly analyzed the nighttime variability of air pollution over Lahore. Gupta et al. [23]conducted a study of Pakistan's major cities (Lahore and Karachi) to investigate the Spatio-temporal distribution of the aerosols. They concluded Lahore to be the most polluted city. Alam et al. [24] similarly analyzed that an increased level of AOD over Pakistan is associated with dust aerosols by using Moderate-resolution Imaging Spectro-radiometer (MODIS) retrieved AOD data. Tariq et al. [25] similarly conducted a study using satellite datasets to analyze aerosol optical properties over the mega city Lahore during the crop residue burning event in October 2013. High values of AOD were observed in Lahore during the burning event.

Angstrom exponent (AE) is a parameter that provides information about the size of aerosol particles by utilizing AOD [26]. AE equal to or greater than 1 indicates the presence of fine-sized aerosols in the air, originating from the burning of biomass and industrial pollution while AE values less than 1 indicate the presence of coarse0sized particles originating from dust [27]. During the monsoon season in 2006, AE was used as an indicator to examine the presence of types of particles over the Arabian Sea and the Bay of Bengal [28].

The article "Seasonal correlation of aerosols with soil moisture, evapotranspiration, and vegetation over Pakistan using remote sensing" was retracted in 2024. Reasons: unreliable results or conclusions; a breach of policy by an author; concerns about the authorship.

Singh et al. [29] studied the variation of aerosols and their size distribution over India and observed the dominance of fine-mode aerosols. Similarly, Tariq and ul-Haq [30] reported a high value of AE in January and a low one in July from 2006 to 2010 over a mega city of Pakistan (i.e. Lahore). In the past, to have an understanding of aerosol trends, different sensors have been used including, “Advanced Very High-Resolution Radiometer (AVHRR)”, “Ozone Monitoring Instrument (OMI)”, “Multiangle Imaging Spectro-Radiometer (MISR)” and “Sea-viewing Wide Field of view Sensor (SeaWiFS)” [21,[31], [32], [33], [34]].

Densely vegetative areas have a significant impact on wind speed (WS) and adhere to the movement of pollutants over a long distance from the ground [35]. Sakar and Kafatos [36] conducted a similar study on the effects of meteorological parameters on aerosols over the northern Indian subcontinent. The following researchers [37,38] conducted a study in Pakistan to examine the association of aerosols with “enhanced vegetation index” and several different meteorological parameters from which they found a positive effect of enhanced vegetation index on aerosols. On the other hand, Chakraborty et al. [39] analyzed the effects of aerosols on the growth of trees during the growing season and they found a positive effect to be present. Gerstl and Zardecki [40] carried out a study to examine the indirect effect of aerosols on plant life. Tariq et al. [38] carried out a study to investigate the relationship of aerosols with enhanced vegetation index and meteorological parameters in Pakistan.

Previously conducted studies have investigated the spatiotemporal distribution of aerosols emitted from anthropogenic activities over Pakistan [10,25,30,[41], [42], [43]]. According to our knowledge, no study has so far been conducted to analyze the relationship of aerosols with SM, evapotranspiration, normalized difference vegetation index (NDVI), and meteorological parameters during different seasons. Therefore, this study aims to investigate seasonal variations of AOD and AE and their relationship with SM, evapotranspiration, NDVI, and meteorological parameters (i.e WS, surface temperature, precipitation, and relative humidity) using long-term data from 2002 to 2022 over Pakistan.

## 2 Site description and methodology

### 2.1 Study area

Pakistan is a densely populated country having a population of 225 million. It is located between latitudes 24°–37° N and longitude 61°–76° E. There lies the Himalaya and Karakoram ranges in the northern areas of Pakistan (as shown in Fig. 1). However, plains exist along with river Indus in the center which is a very important for agricultural purposes [44].

The article "Seasonal correlation of aerosols with soil moisture, evapotranspiration, and vegetation over Pakistan using remote sensing" was retracted in 2024. Reasons: unreliable results or conclusions; a breach of policy by an author; concerns about the authorship.

**Fig. 1:** Elevation map of Pakistan showing different provinces.

In this study, we have selected all the provinces of Pakistan i.e., Punjab, Sindh, Baluchistan, and Khyber-Pakhtunkhwa. These provinces are selected based on different climatic conditions. Details of each province with the source of aerosols are discussed in Table 1. Punjab lies in the eastern region of Pakistan, a densely populated and industrialized area. Khyber-Pakhtunkhwa lies in the northern region of Pakistan which is rich in mineral deposits and is less urbanized due to hilly topography. Baluchistan is a less populated province due to its arid climate, and it is located in the western region of Pakistan while the province of Sindh lies in the southern region of Pakistan, and is relatively densely populated due to industrialization.

**Table 1:** Spatial bounding of provinces in Pakistan along with the anthropogenic sources of aerosols. Koppen – Geiger climate classification based on precipitation, vegetation, and seasonality in provinces of Pakistan [45].

Provinces	Spatial bounding	Climate Classification and population density	Notable sources of aerosols
**Punjab**	70° 18′ 45" −27° 56′ 57.12″ E, 75° 35′ 9.24″-33° 45′ 0″N	Hot semi-arid area (BSh) having a high-density population.	Rice and wheat residue burning during pre- and post-monsoon, megacities (Lahore, Faisalabad), and power plants.
**Sindh**	65° 44′ 31.92″-23° 54′ 22.68″ E, 72° 46′ 24.24"-29° 10′ 46.92″N	Hot desert climate (BWh) along with the highly dense population.	Gawadar and Chahbar ports activities, burning of fossil fuels, dust/sand from the desert of Thar and Cholistan.
**Baluchistan**	59° 56′ 29.04″-25° 18′ 45″ E, 69° 57′ 39.24″-32° 20′ 37.68″N	Warm desert (BWh), less densely populated area.	Mining activities and sand dust.
**Khyber Pakhtunkhwa**	68° 22′ 44.04″-32° 20′ 37.68″ E, - 73° 18′ 2.88″ 37° 37′ 1.92″ N	Humid subtropical climate (Cfa), moderately populated.	The coal is used for home heating during the winter season, dung burning, and forest fires.

### 2.2 Data sets

#### 2.2.1 AOD and AE

In 1999, MODIS sensor onboard the Aqua satellite was launched [46]. It has 36 spectral bands along with high radiometric resolution at 12 bits to monitor aerosols, cloud cover, and daily global radiation budget[47]. For retrieval of aerosols over the land and ocean, two different algorithms are used; the deep blue and dark target [47]. In our study, we have used a monthly product of MODIS-Aqua retrieved data of combined dark target and deep blue AOD at 0.55 μm (MYD08_M3v6.1) with 1° × 1° spatial resolution from NASA's Giovanni website (https://giovanni.gsfc.nasa.gov/giovanni/). Similarly, for AE, we have used MODIS-Aqua with deep blue Angstrom Exponent for land (0.412–0.47 μm) monthly product (MYD08_M3v6.1) with 1° × 1° spatial resolution from the same website. Version 6 of AOD and AE is the latest and most improved product that provides improved cloud masking and atmospheric profile algorithms.

The article "Seasonal correlation of aerosols with soil moisture, evapotranspiration, and vegetation over Pakistan using remote sensing" was retracted in 2024. Reasons: unreliable results or conclusions; a breach of policy by an author; concerns about the authorship.

#### 2.2.2 PR, SM, evapotranspiration, NDVI, SWS, RH, and AT

Data for a meteorological and topological parameter was obtained from Atmospheric Infrared Sounder (AIRS) for Relative Humidity (RH) at 925 hPa. Similarly, data for PR, NDVI, surface wind speed (SWS), and Atmospheric temperature (AT) was obtained from the Tropical Rainfall Measuring Mission (TRMM), MODIS sensor onboard the Terra satellite and the Modern-Era Retrospective analysis for Research and Applications, version 2 (MERRA-2) Model respectively. Data for SM and evapotranspiration was collected from Global Land Data Assimilation System (GLDAS). All the datasets are collected from the website Giovanni NASA (https://giovanni.gsfc.nasa.gov/giovanni/). Details of all the datasets are given in Table 2.

**Table 2:** Details of the dataset used in this study.

Product name	Sensor/model	Retrieval time (day/night)	Spatial resolution (degrees)	Product name/version/level	Units
AOD (MYD08_M3 v6.1)	MODIS-Aqua	Daytime	1° × 1°	Version 6/level 3	Unit less
AE (MYD08_M3 v6.1)	MODIS Aqua	Daytime	1° × 1°	Version 6/level 3	Unit less
Precipitation Rate (TRMM_3B43_v7)	TRMM	Daytime	0.25° × 0.25°	Version 7/level 3	mm/day
Surface wind speed (M2TMNXFLX v5.12.4)	MERRA-2 Model	Daytime	0.5° × 0.625°	Version 5	ms^−1^
Relative Humidity (AIRS3STM v6.0)	AIRS	Daytime	1° × 1°	Version 7/level 3	Percent
Surface Temperature (FLDASNOAH01CGLMOO1)	FLDAS	Daytime	1° × 1°	Version 6/level 3	kelvin
NDVI (MOD13C2v006)	MODIS- Terra	Daytime	0.5° × 0.5°	Version 6/level 3	NDVI
Soil moisture content (GLDAS_NOAHO25_Mv2.1)	GLDAS	Daytime	0.25°	Version 2	kgm^−2^
Evapotranspiration (GLDAS_NOAHO10_Mv2.1)	GLDAS	Daytime	0.25°	Version 2	kgm^−2^S^−1^

### 2.3 Methodology

We have downloaded data of AOD and AE from the year 2002–2021 during different seasons; winters (December, January, February), spring (March, April, May), summer (June, July, August), and autumn (September, October, November). These datasets were utilized to observe the spatial variability of AOD and AE over different seasons among all provinces of Pakistan.

Furthermore, seasonal datasets were also downloaded for NDVI, SM, evapotranspiration, and other meteorological parameters. Data was downloaded in the form of TIFF (tagged image file format) and later on, imported into the ArcGIS software.

The article "Seasonal correlation of aerosols with soil moisture, evapotranspiration, and vegetation over Pakistan using remote sensing" was retracted in 2024. Reasons: unreliable results or conclusions; a breach of policy by an author; concerns about the authorship.

ArcGIS software was used to carry out all the analysis. After downloading the data, the resolutions of the data sets were equalized by using a resampling tool in the data management category of ArcGIS. Finally, correlation maps were exported from the ArcGIS software, and the results were compared.

## 3 Results and discussion

### 3.1 Spatial distribution of AOD and AE in Pakistan

Fig. 2 presents the spatial distribution of AOD and AE over all provinces of Pakistan. The higher values of AOD were observed in Punjab (0.55) and Sindh (0.48) during the study period, which extended into the southern region. Desert dust transported from Thar and Cholistan deserts is the major source of AOD contribution over Punjab and Sindh. High AOD values in Punjab and Sindh are also associated with rapid urbanization, biomass burning, crop residue burning, along with desert dust transported from Thar and Cholistan deserts. Our finding is supported by Tariq and Ali [48], who analyzed that the increase in the flux of aerosols in the regions of Punjab and Sindh is contributed by dust and desert aerosols transported from Thar and Cholistan deserts through the wind. Also, Zhang et al. [21] and Zhang et al. [49] similarly pointed out high AOD values in the southern region of Pakistan (including Sindh, and Baluchistan) due to rapid increases in population, industry, and urbanization. Khan et al. [21] similarly indicated the dominance of sea salt transported from the Arabian Sea over Karachi from 2004 to 2021. Ashraf et al. [44] pointed out that Punjab had the highest aerosol loading which badly impacted the visibility of Punjab. Similarly, low values of AOD (approximately 0.23) were observed in Khyber Pakhtunkhwa which lies in the northwestern region of Pakistan. Alam et al. [24] reported that northern western areas of Pakistan experience less flux of AOD due to less population and more agricultural land.

**Fig. 2:** Spatial distribution of (a) AOD and (b) AE in Pakistan.

By contrast, AE distribution among provinces of Pakistan was in such a way that the approximate values of 1.06, 1.15, 0.89, and 0.82 of AE are observed in the eastern, northern, southern, and western regions of Pakistan respectively. Variation of AE was high in Punjab and Khyber Pakhtunkhwa (approximately 1.06 and 1.15), indicating that the fine mode aerosol particles increase in these regions. The dominance of fine-mode aerosols in Khyber Pakhtunkhwa and Punjab indicated an increase in biomass burning and related anthropogenic activities, especially in winter. Ali et al. [42] analyzed the properties of aerosols in Pakistan and showed the dominance of coarse and fine mode particles over Punjab respectively. Dust from the Sahara and Thar regions is the major source of coarse-mode particles over Sindh. Similarly, our study showed elevated values of AE for Khyber Pakhtunkhwa and Punjab while a lower value of AE for Sindh and Baluchistan. So, the variability of AOD and AE in all four provinces of Pakistan as illustrated in Fig. 2 indicates that high AOD values are associated with anthropogenic activities and dust particles transported from desert regions. Low AE values in Sindh as that of Punjab indicating the dominance of coarse mode are associated with desert dust transported from Thar and Sahara regions.

The article "Seasonal correlation of aerosols with soil moisture, evapotranspiration, and vegetation over Pakistan using remote sensing" was retracted in 2024. Reasons: unreliable results or conclusions; a breach of policy by an author; concerns about the authorship.

#### 3.1.1 Seasonal variation of AOD

Fig. 3 illustrates that AOD peaked during the summer and autumn seasons, while remained low in spring and winter in all provinces of Pakistan. In spring, peak values were found to be in Punjab (0.45) and Sindh (0.43). Further, an increasing trend for AOD was recorded in summers for all provinces of Pakistan with peak values in Punjab (0.8) and Sindh (0.7). In the spring and winter season, AOD decreased significantly across all the provinces of Pakistan with the highest value for spring (0.54) and approximately 0.48 for winter. These seasonal variations indicated that in summers severe aerosol extinction events occurred. Higher AOD values in summers in Punjab (0.84) and Sindh (0.84) are attributed to various anthropogenic activities such as industrial and fossil fuel burning, several open burning sources, smoke coming from forest fires, and water-soluble agricultural aerosols [50]. Khan et al. [21] similarly noted the high value of absorbing aerosols over Pakistan in the summer season from October 2004 to December 2021.

**Fig. 3:** Seasonal variation of AOD in (a) Winter, (b) Summer, (c) Spring, (d) Autumn in Pakistan.

#### 3.1.2 Seasonal variation of AE

The seasonal spatial distribution of AE from 2002 to 2022 is shown in Fig. 4. AE is an indicator for the size distribution of aerosols. High spatial AE variability was observed in the winter season over Punjab (1.3), Khyber Pakhtunkhwa (1.2), Sindh (0.5), and Baluchistan (0.4). Similarly, in spring the highest value of AE was in Khyber Pakhtunkhwa (1.6) followed by Punjab (0.4), Sindh (0.3), and Baluchistan (0.4). During summers, the AE value was highest for Khyber Pakhtunkhwa (1.8) followed by Punjab (1), Sindh (0.8), and Baluchistan (0.6). For autumn the highest value for AE was in Khyber Pakhtunkhwa (1.5) followed by Punjab (1.4), Sindh (0.8–0.4), and Baluchistan (0.8–0.4). These results indicated that the value of AE remained above 1 throughout all the seasons in Khyber Pakhtunkhwa followed by the highest value in Punjab (approximately 1.3), especially in winter. In the study of Simpson et al. [51] and Kaskaoutis et al. [52] the authors found that the burning of wood is the cheapest source of getting heat so the concentration of fine-mode aerosols increases. People survive by burning wood that contributes to biomass aerosols. Several other studies also confirm the fact that the burning of wood, dung, and coal in winter contributes to fine aerosol particles [42].

The article "Seasonal correlation of aerosols with soil moisture, evapotranspiration, and vegetation over Pakistan using remote sensing" was retracted in 2024. Reasons: unreliable results or conclusions; a breach of policy by an author; concerns about the authorship.

**Fig. 4:** Seasonal variation of AE during (a) Winter, (b) Summer, (c) Spring, (d) Autumn in Pakistan.

#### 3.1.3 Seasonal variation of NDVI

Fig. 5 shows the seasonal variation of NDVI during the winter season. Punjab (0.6) and a few areas of Sindh (0.6), and Khyber Pakhtunkhwa (0.3) show moderate values of NDVI. However, in the summer, the areas of Kashmir (0.8) and northern Khyber Pakhtunkhwa (0.8) show the highest values of NDVI. Similarly, in the spring season Punjab (0.7) southern Kashmir (0.8), and northern Khyber Pakhtunkhwa (0.8) show the highest values of NDVI. In the autumn season, Punjab (0.6), a few areas of Sindh (0.6), northern Khyber Pakhtunkhwa (0.7), and southern Kashmir (0.7) show the highest NDVI. Whereas Baluchistan (0.2) and some areas of Kashmir (0–0.1) have the lowest NDVI throughout all the seasons.

**Fig. 5:** Seasonal variation of NDVI in (a) Winter, (b) Summer, (c) Spring, (d) Autumn in Pakistan.

#### 3.1.4 Seasonal variation of wind speed

According to Fig. 6, the highest WS is found in the areas of Baluchistan (10–12 km/h) during the winter and spring seasons. Similarly, high WS is found in Sindh (12 km/h) during the spring season. During the summer season, WS is found to be lower (1–3 km/h) in areas of northern Khyber Pakhtunkhwa (1–3 km/h), Punjab (3 km/h), and a few areas of Sindh (4 km/h). During the summer season, it is found to be 5–6 km/h in Baluchistan.

**Fig. 6:** Seasonal variation of WS during (a) Winter, (b) Summer, (c) Spring, (d) Autumn in Pakistan.

#### 3.1.5 Seasonal variation of temperature

Temperature is also one of the major natural factors affecting the scattering of pollutants in the atmosphere. It can be seen in Fig. 7 that temperature is found to be high in the areas of Punjab (300–320 k) and Sindh (300 k) during all seasons. Baluchistan (310–320 k) has the highest value of temperature during the summer and autumn seasons. Low temperature is found in the area of Kashmir (240–260 k) in all seasons. As the temperature increases, the moisture in the atmosphere decreases resulting in scattering of aerosols in the atmosphere. Khan et al. [21] similarly observed a positive correlation of UVAI with temperature in Pakistan from 2004 to 2021.

The article "Seasonal correlation of aerosols with soil moisture, evapotranspiration, and vegetation over Pakistan using remote sensing" was retracted in 2024. Reasons: unreliable results or conclusions; a breach of policy by an author; concerns about the authorship.

**Fig. 7:** Seasonal variation of temperature in (a) Winter, (b) Summer, (c) Spring, (d) Autumn in Pakistan.

#### 3.1.6 Seasonal variation of RH

According to Fig. 8, the RH is found to be highest in northern Khyber Pakhtunkhwa (70%) and Kashmir (70%) areas during the winter and spring seasons. Similarly, moderate (30–45%) RH is found in Sindh, Punjab, and Khyber Pakhtunkhwa during the summer and autumn seasons. The lowest values (10–20%) of RH are found in Baluchistan during all the seasons. As the moisture in the atmosphere increases the visibility in the atmosphere decreases because of the increase in the concentration of absorbing aerosols in the atmosphere [21].

**Fig. 8:** Seasonal variation of relative humidity in (a) Winter, (b) Summer, (c) Spring, (d) Autumn in Pakistan.

#### 3.1.7 Seasonal variation of precipitation

According to Fig. 9 the highest values for the PR are found in northern Khyber Pakhtunkhwa (0.8 mm/day), near Quetta (0.4 mm/day), and southern Kashmir (0.8 mm/day) during the winter season. Similarly, in the spring season PR is found to be moderate to high in Khyber Pakhtunkhwa (0.1 mm/day). During the summer and autumn seasons, low to moderate precipitation is found in northern Punjab (0.1 mm/day) and Khyber Pakhtunkhwa (0.1 mm/day). However, in all seasons precipitation remained moderate (0.02–0.1 mm/day) in Punjab and lowest (0.02–0.05 mm/day) in Baluchistan.

**Fig. 9:** Seasonal variation of precipitation in (a) Winter, (b) Summer, (c) Spring, (d) Autumn in Pakistan.

#### 3.1.8 Seasonal variation of SM

According to Fig. 10 SM remained low to moderate (120-150 kgm^−2^) during all seasons in Baluchistan, Khyber Pakhtunkhwa, and some areas of Sindh. The lowest range of SM content (40-60 kgm^−2^) is found majorly in Punjab and Sindh. Similarly, the highest SM content (280 kgm^−2^) is found to be in northern Kashmir.

**Fig. 10:** Seasonal variation of soil moisture (SM) in (a) Winter, (b) Summer, (c) Spring, (d) Autumn in Pakistan.

#### 3.1.9 Seasonal variation of evapotranspiration

According to Fig. 1S, in winter and summer seasons, the lowest evapotranspiration rate is found over Baluchistan (3.9 × 10^−0.07^), Sindh (3.9 × 10^−0.07^), and southern eastern Punjab (6.7 × 10^−0.06^). However, a moderate evapotranspiration rate is observed in northern Punjab (1.5 × 10^−0.05^) during winter. In summer, a high rate of evapotranspiration (4.7 × 10^−0.05^) is found in northern Punjab, all over Khyber Pakhtunkhwa, and in southern Kashmir. Similarly, in the case of Kashmir, a high rate of evapotranspiration (4.7 × 10^−0.05^) is found during the spring and autumn seasons. A moderate range (3.5 × 10^−0.06^) of evapotranspiration is found in Punjab, Khyber Pakhtunkhwa, and in some cities of Sindh during the autumn and spring seasons. Similarly, the lowest value (3.9 × 10^−0.07^) is found in Baluchistan during the autumn and spring seasons.

The article "Seasonal correlation of aerosols with soil moisture, evapotranspiration, and vegetation over Pakistan using remote sensing" was retracted in 2024. Reasons: unreliable results or conclusions; a breach of policy by an author; concerns about the authorship.

### 3.2 Seasonal correlation of AOD with AE, NDVI, SM, evapotranspiration, and meteorological parameters

The correlation between AOD and AE derived from Aqua-MODIS over Pakistan has been shown in Fig. 2S. During the winter season, a very weak positive correlation can be observed in Punjab (∼0.4), Sindh (∼0.2), and in some areas of Baluchistan (∼0.1). According to Fig. 4, Fig. 5 high burden of fine-mode aerosols is present in these regions due to industrial and biomass burning [53]. Similarly, a strong negative correlation between AOD and AE can be observed in Baluchistan (0.2). According to Fig. 4, Fig. 5, a high value of AOD (0.9) and a low value of AE (0.8) in these regions indicate the presence of coarse-mode aerosols especially dust aerosols [38]. During the summer season, a weak positive correlation between AOD and AE has been observed in Khyber Pakhtunkhwa, Punjab, and Sindh. AOD is higher (1.2) during the summer season followed by a high value of AE (1.2) (Fig. 4, Fig. 5) indicating the presence of a high burden of aerosols having fine particle size. Similarly, a strong negative correlation (−0.2) is observed between AOD and AE in Baluchistan and a few areas of Kashmir. These areas have a high aerosol burden but a low value of AE indicating the presence of coarse mode particles. Tariq et al. [50] conducted a similar study in which they reported that Baluchistan has high AOD due to high temperatures in summer and high dust storm frequency.

During the spring season, a very weak positive correlation has been observed in northern Khyber Pakhtunkhwa, Kashmir, and Punjab. These areas have an AOD value of ∼0.7 with the presence of coarse mode particles indicated by a low value of AE (0.6) (Fig. 4, Fig. 5) except for in Khyber Pakhtunkhwa where burning coal in the spring season produces fine mode particles. Tariq et al. [38] conducted a similar study in which they reported that Khyber Pakhtunkhwa experiences a high burden of fine-mode aerosols in spring due to the burning of coal and crop residue. Similarly, a strong negative correlation can be observed in Baluchistan (∼−0.4) and some areas of Sindh (∼−0.5). A negative correlation during the spring season validates the presence of coarse mode particles (0.8) followed by low aerosol burden (AOD = 0.6) (Fig. 4, Fig. 5). Increased traffic and industries are responsible for the contribution of dust in the atmosphere of Sindh [54]. Moreover, during the autumn season, a strong positive correlation can be observed in Punjab (∼0.6) and in a few areas of Sindh. A strong positive correlation indicates the presence of a high burden of aerosols followed by the presence of a fine and mixed type of aerosols indicating a high value of AE (Fig. 4, Fig. 5). This season shows the prevailing dust aerosols over industrial, biomass, and urban aerosols [42]. Similarly, a strong negative correlation has been observed in Baluchistan and in some areas of Khyber Pakhtunkhwa that indicates a low aerosol burden [49].

The article "Seasonal correlation of aerosols with soil moisture, evapotranspiration, and vegetation over Pakistan using remote sensing" was retracted in 2024. Reasons: unreliable results or conclusions; a breach of policy by an author; concerns about the authorship.

Fig. 3S shows a strong positive correlation of AOD with NDVI in the western regions of Punjab (∼0.7) and southern Khyber Pakhtunkhwa (∼0.8) during the winter season. From Fig. 3, Fig. 5, it can be seen that in Khyber Pakhtunkhwa the aerosol burden is low (0.2) and NDVI has a moderate value (∼0.4) whereas in Punjab aerosol burden is moderate (0.7) and NDVI is higher. Vegetation plays an important role in modifying the movement of aerosols [55]. Despite the high NDVI in Punjab, smoke from traffic and industries contributes to the aerosol burden due to dense fog in winter [56]. Similarly, a strong negative correlation can be observed in Baluchistan, especially in areas of Gwadar, Quetta, and Zhob along with some cities in western Khyber Pakhtunkhwa and southern Sindh. Aerosol burden is found to be low in winter in Baluchistan as well as in southern Sindh and western Khyber Pakhtunkhwa due to low levels of vegetation. During the summer season, a weak positive correlation can be seen in Khyber Pakhtunkhwa and western Punjab. Punjab has a high urbanization rate that reduces the vegetation index [57]. A negative correlation can be observed in Kashmir (0.7) where the aerosol burden is found to be low (0.4) because the NDVI level is high (0.8) (Fig. 3, Fig. 5). Mountainous areas play a great role in acting as a barrier for aerosol dispersal [58].

During the spring season, a weak positive correlation between NDVI and AOD can be observed in Khyber Pakhtunkhwa. According to Fig. 3, Fig. 5, the NDVI level is low (0.3–0.5), and the aerosol burden is moderate (0.6) in Khyber Pakhtunkhwa. Similarly, a medium negative correlation can be observed in the area of Baluchistan (−0.1), southern Punjab (0), and Kashmir (−0.1) which includes cities like Zhob (−0.1), and Quetta (−0.1). According to Fig. 3, Fig. 5, the aerosol burden is low (0.1–0.4) in the areas of Punjab (0.3), Baluchistan (0.3), and Kashmir, and the NDVI index is also low (0.4) in the above-mentioned areas except for in Kashmir (0.7). The vegetation index is found to be very low in Baluchistan because it is a deserted area and receives very less rainfall [59]. Punjab is found to have a rapid rate of urbanization and a high rate of industrialization which leads to an increase in land use over there [60,61]. Similarly, during the autumn season, a strong positive correlation between AOD and NDVI can be observed in Khyber Pakhtunkhwa (0.8) and northern Baluchistan (0.7). According to Fig. 3, Fig. 5, in Khyber Pakhtunkhwa NDVI is moderate (0.4–0.6) and the aerosol burden is low (0.2). However, in Baluchistan aerosol burden (0.3) and NDVI (0.2), both are low due to less rainfall and low WS in northern Baluchistan which causes less dispersal of aerosols in the region [62]. A strong negative correlation can be observed in western Baluchistan (−0.1) in Fig. 3S. It can be observed in Fig. 3, Fig. 5, that western Baluchistan has low NDVI (0.1) and moderate aerosol burden (0.7). Western Baluchistan faces severe evapotranspiration that makes the air less humid contributing to a reduction in vegetation [63]. All these results show that an increase in NDVI decreases aerosol dispersal and a decrease in NDVI increases aerosol dispersal, so these two parameters have an indirect relation in all seasons except for in spring and autumn.

The article "Seasonal correlation of aerosols with soil moisture, evapotranspiration, and vegetation over Pakistan using remote sensing" was retracted in 2024. Reasons: unreliable results or conclusions; a breach of policy by an author; concerns about the authorship.

According to Fig. 4S, during winter weak positive correlation can be observed in the northwestern regions of Baluchistan. We can observe a weak negative correlation between AOD and WS in northeastern Punjab where the aerosol burden is found to be higher (0.8) and WS is lower (3 km/h). Smog episodes in Punjab hold the aerosols in the atmosphere and have a low speed of wind []. Nicolaou [64] showed in their study that WS in the atmosphere settles down aerosols on the land under the action of gravity. During the summer season, a weak positive relationship between WS and AOD is observed in the area of Kashmir (Fig. 4S). Similarly, a negative correlation can be observed in northern Baluchistan including the cities of Quetta, Zhob, Khuzdar, and the southern region of Khyber Pakhtunkhwa. Slow winds in northern Baluchistan and southern Khyber Pakhtunkhwa due to low to moderate temperature causes relatively weak vertical convection thus having low aerosol burden [65].

During the spring season, a strong positive correlation is observed in southern Punjab, almost all the areas of Sindh, and a few areas of Baluchistan. The aerosol burden is found to be moderate (0.7) in respective areas in Punjab, Sindh, and Baluchistan. Similarly, WS is also moderate (greater than 6 km/h). An extremely weak negative correlation is found in northern Punjab. In spring, the aerosol burden is found to be moderate because frequent dust storm events occur in which wind helps to transport the aerosols from Thar, Thal, and surrounding arid areas to Sindh, Baluchistan, and Punjab [66,67]. The temperature in northern Punjab is low to moderate in spring due to which aerosol burden is low.

The article "Seasonal correlation of aerosols with soil moisture, evapotranspiration, and vegetation over Pakistan using remote sensing" was retracted in 2024. Reasons: unreliable results or conclusions; a breach of policy by an author; concerns about the authorship.

During the autumn season (Fig. 4S) positive relationship between AOD and WS is found in the areas of southwestern Baluchistan and almost in the whole of Sindh. According to Fig. 3, Fig. 6, aerosol burden (AOD = 0.4) and WS (9 km/h) both are low in these regions. Similarly, a strong negative relation is observed in Baluchistan and southern Khyber Pakhtunkhwa. According to Fig. 3, Fig. 6, aerosol burden (∼0.3) and WS (3 km/h) are both low. Pakistan faces low AOD during post-monsoon due to fewer dust storms in this season and low windspeed does not allow the movement of aerosols.

From Fig. 5S, it can be seen that during the winter season, a weak positive correlation is observed between AOD and temperature in western southern Baluchistan. RH remains low in desert areas so, fewer aerosols are present in the respective area at low temperatures, especially in Baluchistan [68]. Ramachandran and Cherian [69] conducted a study that showed that Kashmir has a relatively lower annual AOD because of less traffic and less industrialization as compared to other areas.

A weak negative correlation is found to be in northern Khyber Pakhtunkhwa. Aerosols are found to be moderate in concentration (0.6) but the temperature is also low to moderate (180 k) (Fig. 4, Fig. 8). Tariq et al. [38] conducted a similar study in which AOD is moderate to high because people burn wood, biomass, and coal to overcome cold in winter and for cooking purposes in Khyber Pakhtunkhwa.

During the summer season, a weak positive correlation is found in western Baluchistan, Sindh, southeastern Punjab, and Khyber Pakhtunkhwa. According to Fig. 3, the aerosol burden is higher (greater than 1) in Sindh and Punjab. However, in Baluchistan, the aerosol burden is moderate to high (0.8) along with the moderate temperature. During summers SM is a deficit in Baluchistan and a drought situation occurs that enhances the aerosol burden over there [59]. Similarly, Fig. 7 shows a negative relationship of AOD with temperature which is found in northwestern Punjab and southwestern Khyber Pakhtunkhwa. Also, Tariq et al. [70] and ul-Haq et al. [71] conducted a study in Pakistan in which they found out that in summer high AOD is due to an increase in anthropogenic activities i.e., road dust, smoke, dust from heavy machines, and burning of crops. Aerosols generated from human activities affect the climate by scattering and absorbing the solar radiation reaching the earth [72]. Khan et al. [21] similarly observed a strong positive correlation of UVAI with temperature throughout Pakistan from 2004 to 2021.

The article "Seasonal correlation of aerosols with soil moisture, evapotranspiration, and vegetation over Pakistan using remote sensing" was retracted in 2024. Reasons: unreliable results or conclusions; a breach of policy by an author; concerns about the authorship.

During the spring season, a strong positive correlation between AOD and temperature is found in Sindh, Baluchistan, and southern Khyber Pakhtunkhwa. Similarly, a negative correlation is found in Khyber Pakhtunkhwa and Kashmir. During the autumn season, a strong positive correlation is found all over Baluchistan, and Khyber Pakhtunkhwa which includes Chagai, Zhob, Quetta, Khuzdar, Peshawar, Mardan, and Kohistan. AOD is lowest during the spring, winter, and autumn seasons in above mentioned regions because of weak vertical mixing in the atmosphere and the absence of strong connective winds in the low temperatures [68].

A negative correlation is observed in southern western Punjab and Gilgit Baltistan. Punjab has high AOD due to the harvesting season of rice in which rice husk contributes to atmospheric pollution in the atmosphere followed by the burning of left-over rice residues [73]. All the above discussion shows that AOD and temperature have a direct relationship between them in all seasons. An increase in temperature increases the aerosol burden and vice versa.

According to Fig. 6S, during the winter season, a positive correlation (0.7) is found in northwestern Baluchistan and Khyber Pakhtunkhwa. According to Fig. 3, Fig. 8, both RH (greater than 20%) and AOD (0.3) are low in the above-mentioned areas of Pakistan. A weak negative correlation is found in Baluchistan (−0.5) and Sindh (−0.4). The RH is found to be low (20%) along with a low aerosol burden (0.2) (Fig. 3, Fig. 8). Low RH in winter along with low temperatures does not trap aerosols in the atmosphere thus reducing the aerosol burden in the atmosphere.

During summers, a positive correlation is found in northwestern Punjab (0.8) and in Khyber Pakhtunkhwa (0.9). A moderate (40%) amount of RH is present in the above regions with low AOD (0.6) in Khyber Pakhtunkhwa and moderate to high AOD (greater than 0.8) in Punjab. A negative correlation is found in some areas of Punjab (−0.6), Sindh (−0.6), and Gilgit Baltistan (−0.7). However, the cities of Srinagar, Muzaffarabad, and Gilgit have a low aerosol burden (0.3) and moderate RH (50%) (Fig. 4, Fig. 9). Moderate to high RH in summers intensifies the hygroscopic growth of aerosols along with the gas-to-particle conversion process thus increasing AOD [74]. Northern mountainous areas have suppressed aerosol inflow than the southern areas because of topography, less human activities, decreases in atmospheric pressure, and wind advection [75]. These are the reasons that despite having moderate humidity aerosol burden is low in Muzaffarabad and Srinagar.

The article "Seasonal correlation of aerosols with soil moisture, evapotranspiration, and vegetation over Pakistan using remote sensing" was retracted in 2024. Reasons: unreliable results or conclusions; a breach of policy by an author; concerns about the authorship.

During spring, a strong positive correlation is found in south-eastern Sindh (∼1) and Kashmir (∼0.7). According to Fig. 3, Fig. 8, RH is low in Sindh (25%) and high in Kashmir (60%) whereas AOD is high (0.8) in Sindh and low in Kashmir (0.2).

A negative correlation is found in southern Khyber Pakhtunkhwa (−0.7), and Baluchistan (−0.8). The RH is low (30%) in these areas along with a low AOD (0.3). During autumn, a strong positive correlation is found in a few areas of Khyber Pakhtunkhwa (1), northern western Punjab (0.8), eastern Baluchistan (0.7), and all over Sindh (greater than 0.8). Areas of Peshawar and Khuzdar show relatively low aerosol burden (0.2) with low to moderate (35%) RH. However, in Sindh and Punjab, the aerosol burden is high (greater than 0.9) and RH is low (<20%). A negative correlation is found in northwestern Baluchistan (∼-1) so, according to Fig. 3, Fig. 8 aerosol burden is low (0.2) along with less RH (20%). During the spring season, agricultural harvesting and biomass burning along with emissions from industries is the largest source of increase in aerosol burden. High WS during the autumn season helps in the transportation of aerosols thus increasing the aerosol burden [76].

All these results show that AOD and RH show a direct relation in the summer and winter seasons. However, in autumn and spring, AOD and RH show an indirect relationship between them. It can be seen in Fig. 7S that during the winter season, a strong positive correlation of AOD with precipitation is found in northern Baluchistan (0.4) and Khyber Pakhtunkhwa (0.8). According to Fig. 3, Fig. 9, in the winter season aerosol burden is moderate to low (0.2) in Baluchistan and Khyber Pakhtunkhwa whereas, the PR is higher in Khyber Pakhtunkhwa (0.2 mm/day) and low in Baluchistan (0.02 mm/day). The droughted land of Baluchistan lost the majority of SM so, very little evaporation occurs due to which rainfall is very low over there [77,78]. Whereas, in Khyber Pakhtunkhwa aerosol burden is low because precipitation washes out aerosols in the atmosphere. A negative correlation is observed in northeastern Punjab. Punjab has low precipitation (0.02 mm/day) and a high aerosol burden (0.8). The PR is low in Punjab causing a dry climate and short cold season with less humidity. Similarly, the higher rate of vehicular and industrial emissions along with dust and smoke from burning coal contributes to increasing AOD [79].

In summer, a weak positive correlation (0.3) is found in the northern area of Punjab and the eastern area of Khyber Pakhtunkhwa. According to Fig. 3, Fig. 9, these areas have low PR (∼0.02 mm/day) and a high burden of aerosol (0.8). Summers remain a deficit of precipitation especially in eastern Khyber Pakhtunkhwa and Punjab due to the temperature rise which increases the aerosol burden. The fluctuation in PR can be due to various factors such as changes in El Nino and La Nina conditions of the southern Pacific Ocean [80].

The article "Seasonal correlation of aerosols with soil moisture, evapotranspiration, and vegetation over Pakistan using remote sensing" was retracted in 2024. Reasons: unreliable results or conclusions; a breach of policy by an author; concerns about the authorship.

A negative correlation (less than 0.07) is found in a few areas of Punjab, Sindh, and Kashmir. High aerosol burden (1) with low precipitation (0.02 mm/day) is found in Sindh and Punjab. However, in Muzaffarabad, as well as in Srinagar, the aerosol burden is low (0.4), and precipitation (0.2 mm/day) is found to be high to moderate. Precipitation is high in northern Pakistan because it receives winds laden with moisture and rainfall that washes out the aerosols present in the atmosphere [81].

During the spring season, a weak positive correlation is found in a few areas of northeastern Baluchistan, northern Sindh, and Kashmir. These areas have a low PR (0.02 mm/day) and low aerosol burden (0.6) in spring (Fig. 4, Fig. 10). Similarly, a Strong negative correlation (0.06) is found in western Baluchistan. Areas of Baluchistan and Sindh face extreme dry events due to a decrease in rainfall in several years due to climate change and due to a decrease in moisture over the years. Northern areas of Pakistan have a high PR due to humidity, low to moderate temperatures, and high vegetation [62].

During autumn, a strong positive correlation (greater than 0.4) is found in Sindh and Baluchistan. In Sindh, aerosol burden (0.8) is found to be high, whereas precipitation (0.02 mm/day) is found to be low. Similarly, a negative correlation (0.04) is found in Baluchistan and eastern Punjab (Fig. 7S). Significant decrease in evapotranspiration due to the change in the climate of Pakistan due to which temperature keeps on rising results in low precipitation [82]. The increase in AOD over Pakistan can be due to agricultural harvesting, dust storm activities, industrial activities along with economic developments. Ul-Haq et al. [71] conducted a similar study to analyze annual AOD in which they concluded that annual mean AOD was high over Sindh and Punjab followed by Baluchistan, Khyber Pakhtunkhwa, Kashmir, and Gilgit Baltistan. Punjab and Sindh are major economy-producing provinces of Pakistan so this can be the reason for the high AOD. Similarly, in Baluchistan, the Thar Desert is a major reason for a contribution towards high AOD. Ur Rehman et al. [83] pointed out in their study that Indian coal-fired power plants are the major sources that are affecting northeastern Pakistan. Other reasons can be different sources like vehicular emissions, increased industrial emissions, and locally produced dust [24].

The article "Seasonal correlation of aerosols with soil moisture, evapotranspiration, and vegetation over Pakistan using remote sensing" was retracted in 2024. Reasons: unreliable results or conclusions; a breach of policy by an author; concerns about the authorship.

It can be seen in Fig. 8S that during winters, a positive correlation (0.6) can be observed in northern Baluchistan and Khyber Pakhtunkhwa. A negative correlation (−0.3) can be observed over Punjab, Sindh, and southern Baluchistan. According to Fig. 3, Fig. 10, AOD is low (0.4) in Baluchistan and Khyber Pakhtunkhwa and higher (0.9) in Punjab and Sindh whereas SM is moderate (120 kgm^−2^) in Baluchistan and Khyber Pakhtunkhwa and very low (40 kgm^−2^) in Sindh and Punjab. SM is directly linked with precipitation. A decrease in precipitation in Punjab and Sindh during winter ultimately shows a decrease in SM whereas the northern area of Baluchistan, Kashmir, and Khyber Pakhtunkhwa have moderate SM due to low temperature that prevents evapotranspiration and high rainfall that add moisture to the soil. Increased AOD in Punjab and Sindh is due to the low moisture content in the soil [56].

During summers, a positive correlation can be observed in the northern Punjab (0.6) and eastern Khyber Pakhtunkhwa (0.7). Whereas a negative correlation can be observed in southern Punjab (−0.6), northern Khyber Pakhtunkhwa (−0.5), and Srinagar (−0.9). According to Fig. 1, Fig. 4S, AOD is high (0.9) in Punjab and low (0.4) in Khyber Pakhtunkhwa. Whereas SM is low to moderate (120 kgm^−2^) in Khyber Pakhtunkhwa and Srinagar and lowest in Punjab (40 kgm^−2^). During summers SM content in Punjab is low due to the arid climate followed by hot temperatures (above 40 °C) that cause excessive evaporation thus losing moisture from the soil that holds up aerosol [84].

During spring, a weak positive (0.3) correlation can be observed in western Baluchistan and northern Khyber Pakhtunkhwa. Whereas a strong negative correlation (−0.9) can be observed in Sindh and the southern Punjab area. According to Fig. 3, Fig. 10, SM (100 kgm^−2^) and AOD (0.2) both are low in Baluchistan and northern Khyber Pakhtunkhwa. However, AOD is moderate (0.8) in Sindh and Punjab and SM is very low (40 kgm^−2^). SM is low in Baluchistan due to late summer droughts that stress the SM by increasing the evapotranspiration process [77]. Zamin et al. [85] conducted a study in which they reported that swelled and expansive soil followed by desiccation cracks are found in the region of Kohat, Bannu, and Dera Ismail Khan of Khyber Pakhtunkhwa.

During autumn, a strong positive correlation (greater than 0.6) can be observed in Sindh and Baluchistan. Whereas a negative correlation (−0.7) can be observed in western Punjab and the area of Kashmir. According to Fig. 3, Fig. 10, AOD is low (0.4) in Baluchistan and Kashmir. Similarly, AOD is higher in Sindh (0.9) and Punjab (1). SM is low in the above regions due to climate change that makes evapotranspiration excessive leaving behind dry soil. Moreover, AOD is high in Sindh and Punjab due to anthropogenic activities and crop residue burning [70]. All these results prove that AOD and SM have an indirect relationship. An increase in AOD is due to low SM content and a decrease in AOD is due to moderate to high moisture content.

The article "Seasonal correlation of aerosols with soil moisture, evapotranspiration, and vegetation over Pakistan using remote sensing" was retracted in 2024. Reasons: unreliable results or conclusions; a breach of policy by an author; concerns about the authorship.

It can be seen in Fig. 9S that a positive correlation of AOD with evapotranspiration can be observed in Khyber Pakhtunkhwa (0.8), northern Baluchistan (0.7), and western Punjab (0.6), whereas a negative correlation (−0.5) can be observed in eastern Punjab and southern Sindh. According to Fig. 1, Fig. 3S, AOD is low (0.4) in Baluchistan and Khyber Pakhtunkhwa, and higher (0.8) in Sindh and Punjab. Evapotranspiration is low (3.9 × 10^−0.07^ kgm^−2^s^−1^) in Baluchistan, Khyber Pakhtunkhwa, and Sindh. Only Punjab has a high value (4.7 × 10^−0.05^ kgm^−2^s^−1^) for evapotranspiration. Punjab faces high AOD and evapotranspiration due to high temperatures compared to the rest of the provinces. The studies of Shahriar [86] and Kaur et al. [87] have reported in their study that a decrease in rainfall and an increase in temperature have worsened the situation in Punjab by increasing evapotranspiration.

During the summer season, a strong positive correlation (0.9) can be observed in western Punjab and southern Khyber Pakhtunkhwa. Whereas a negative correlation can be observed in Kashmir (−0.6) and southern Punjab (−0.3) (Fig. 9S). According to Fig. 1, Fig. 3S, the AOD burden is high (1.2) in Punjab, however, in Kashmir and Khyber Pakhtunkhwa it is low (0.4). Evapotranspiration is moderate to high in Kashmir, western Punjab, and southern Khyber Pakhtunkhwa (3.9 × 10^−0.05^ kgm^−2^s^−1^) and low in southern Punjab (6.7 × 10^−0.06^ kgm^−2^s^−1^). Rainfall was high over Punjab in monsoon but over a few years, it has moved to northern and western Khyber Pakhtunkhwa due to changes in climatic patterns. A decrease in rainfall in Punjab increases the evapotranspiration rate [62].

During the spring season, a positive correlation can be observed in Kashmir (0.6) and western Khyber Pakhtunkhwa (0.7), whereas a negative correlation (−0.5) can be observed in northern Punjab, Baluchistan, Khyber Pakhtunkhwa, and Sindh. According to Fig. 1, Fig. 3S, the AOD burden is low (0.4) in Punjab, Baluchistan, and Khyber Pakhtunkhwa whereas, in Sindh, AOD remains moderate (0.8). The evapotranspiration rate remains low (2.7 × 10^−0.06^ kgm^−2^s^−1^) in Baluchistan and Sindh but high (4.7 × 10^−0.05^ kgm^−2^s^−1^) in northern Punjab and Khyber Pakhtunkhwa. Similarly, Fig. 9S shows that during the autumn season, a positive correlation (0.9) can be observed in Baluchistan, Khyber Pakhtunkhwa, and Sindh. Whereas a negative correlation can be observed in eastern Punjab (−0.6), western Baluchistan (−0.6), and Srinagar (−0.7). According to Fig. 1, Fig. 3S, AOD is low (0.4) in Baluchistan and Khyber Pakhtunkhwa, moderate (0.7) in Sindh, and high (1) in Punjab. Whereas evapotranspiration is low to moderate (3.5 × 10^−0.05^ kgm^−2^s^−1^) in Baluchistan, Punjab, and Sindh. Khan and Hasan [88] reported in their study that evapotranspiration in Pakistan increases from northern western regions to southeastern regions of Pakistan. Temperature is relatively high in northern Punjab and Khyber Pakhtunkhwa during spring and autumn which plays a role in increasing evapotranspiration. The above results show that AOD and evapotranspiration have an indirect relationship between summer and winter.

The article "Seasonal correlation of aerosols with soil moisture, evapotranspiration, and vegetation over Pakistan using remote sensing" was retracted in 2024. Reasons: unreliable results or conclusions; a breach of policy by an author; concerns about the authorship.

## 4 Conclusion

Environmental pollution is one of the major issues in developing countries like Pakistan. Therefore, in this study, we analyzed aerosol optical properties and their relationship with SM, evapotranspiration, NDVI, and other meteorological parameters over Pakistan from 2002 to 2021. High AOD values observed in Sindh (0.48) and Punjab (0.55) are associated with desert dust and anthropogenic activities within the region. High AE values observed in Punjab (1.06) and Khyber Pakhtunkhwa (1.15) indicate the dominance of fine-mode particles. Furthermore, NDVI was observed to be high (0.8) in Kashmir and Khyber Pakhtunkhwa during winter. Whereas, in Baluchistan (10–12 km/h) and Sindh (12 km/h), WS was observed to be high during the winter and spring season. The correlation of AOD with WS, temperature, SM, and evapotranspiration over Pakistan showed a direct relation whereas, NDVI and precipitation showed an inverse relation throughout the year. Furthermore, during the summer and winter seasons, AOD showed a direct relation to RH. Significant seasonal changes in AOD measurements demand further research into the area's meteorological pollution source location and transportation. Different methods like afforestation, efficient use of fuel, use of public transport, restriction on the use of certain industrial plants, etc. can be used to reduce air pollution.

## Data availability

Data will be made available on request.

## Ethical approval

Not required.

## Consent to publish

Not Applicable.

## Consent to participate

Not Applicable.

## Funding

The work did not receive any funding.

## CRediT authorship contribution statement

**Uzma Basharat:** Conceptualization, Data curation, Formal analysis, Methodology, Software, Writing – original draft. **Salman Tariq:** Conceptualization, Data curation, Formal analysis, Methodology, Software, Writing – original draft. **Muhammad Nawaz Chaudhry:** Conceptualization, Data curation, Formal analysis, Investigation, Software, Writing – original draft. **Muhammad Khan:** Conceptualization, Data curation, Formal analysis, Investigation, Software, Writing – original draft. **Ephraim Bonah Agyekum:** Formal analysis, Investigation, Methodology, Writing – review & editing. **Wulfran Fendzi Mbasso:** Formal analysis, Investigation, Methodology, Writing – review & editing. **Salah Kamel:** Formal analysis, Investigation, Methodology, Writing – review & editing.

The article "Seasonal correlation of aerosols with soil moisture, evapotranspiration, and vegetation over Pakistan using remote sensing" was retracted in 2024. Reasons: unreliable results or conclusions; a breach of policy by an author; concerns about the authorship.

## Declaration of competing interest

The authors declare that they have no known competing financial interests or personal relationships that could have appeared to influence the work reported in this paper.
